# An Intelligent Digital Media Asset Management Model Based on Business Ecosystem

This article has been retracted.

**DOI:** 10.1155/2022/1190538

**Published:** 2022-05-13

**Authors:** Yutong Liu, Peiyi Song

**Affiliations:** School of Economics and Management, Communication University of China, Beijing 100024, China

## Abstract

In the context of media convergence, it is of great significance to study and discuss the intelligent digital media asset management model and build a digital media asset management ecosystem model to carry out effective digital media asset management for media organizations and promote the value creation of digital media content assets. Based on the business ecosystem, this study adopts a system dynamics approach to construct a system dynamics model through theoretical research and simulation analysis. By studying the positioning of intelligent digital media asset management and service patterns, the basic framework of digital media asset management ecosystems is proposed. To explore the interaction between different factors, the system dynamics model of value creation in digital media asset management ecosystems is built in this paper. This study provides new insights for media organizations on building an intelligent digital media asset management model and promoting the development and utilization of media content resources.

## 1. Introduction

Digital media assets refer to the content resources that are owned and controlled by media organizations, with clear copyrights, are stored in digital form, and have economic value. In the convergence media environment, the development and utilization of media content assets are an urgent and important issue for traditional media, involving legal content acquisition, management, transaction, communication, protection, and other links in the industrial chain. Designing and constructing a digital media asset management ecosystem has become the central issue for further promoting media convergence. In the context of media convergence, insisting on “content is king” and researching the ecosystem of digital media asset management are an important measure to promote the integration, diversification, and platform of traditional media and new media. The specific objective of the media platform is to realize media reengineering through the platform, so that the internet-based traditional media can build a new service system through open communication modes and colorful expressions in the convergence media environment, reshape the relationship between users, and achieve sticky connection with users.

At present, our society has entered the era of the digital economy. The core of the digital economy is data, digital technologies, and digital platforms, including the digitalization of content products, services, and links, as well as all economic activities supported by the Internet and digital technologies. With the ever-changing demands of consumers and the emergence of competitors, the updating cycle of content products and services is becoming increasingly faster, which requires media organizations to respond to the market and audience at the fastest speed, formulate new strategies, implement them at the fastest speed, and then make subsequent adjustments. Under the pressure of competition speed, media organizations must integrate resources and develop products through cooperation, analyze audiences' needs with big data technology, and produce diversified innovative content products that meet the needs of different platforms through flexible program production systems. Therefore, in media convergence and digital economy, digital media assets are factors of production and should play a role as a source of competitiveness. Media organizations urgently need to establish an effective digital media asset management ecosystem, so that the new technical system and digital assets can be transformed into efficient productivity output as soon as possible and greatly improve the performance of media organizations.

China's media organizations, represented by radio and television groups, have set up many media asset management systems. After digitization, media content management focused on resource integration, organization, cataloging, access, retrieval, and limited development and utilization. However, the market-oriented content service mode is still immature and lacks resource integration within the industry, collaboration across agencies, and effective business models. Of particular concern is the fact that the existing digital media asset management system has a very limited ability to integrate resources and provide internal and external content services. It not only cannot produce a scale effect but is also not perfect in information docking, value service, cost reduction, rights and interest protection, and other aspects. There is an urgent need to construct the management mode of digital media assets from the perspective of business ecosystems and address the related problems to further integrate and develop the massive digital media assets. Therefore, based on the business ecosystem, this study first expounds on the positioning of the digital media asset management mode and service patterns. Then, the system dynamics approach was used to construct a digital media asset management ecosystem model, and the value creation process of media content was studied. The dynamic evolution process of influencing factors of content asset transfer between media organizations is considered. It is hoped that this research will contribute to a deeper understanding of managing digital media assets effectively and achieving a greater value of content assets for media organizations.

Moore, who raised the business ecosystem, believes that the business ecosystem is an economic union based on the interaction between organizations and individuals, producing products and services valuable to consumers. The basic idea of a business ecosystem is to emphasize the connection and interdependence of participants in economic activities with common goals. Through the cooperation of many enterprises in a symbiotic relationship, business ecosystems can create the value of a single enterprise that cannot be created [1]. This can provide timely access to develop new knowledge and technologies outside the organization, allowing the organization to focus on its core competence and allowing the partners to better use other areas of expertise and resources. This is critical to competitive success in high-tech industries [2]. There is a growing body of literature that recognizes that the key to gaining competitive advantages in the process of coevolution is the innovation process of an organization by cocreation enhancement [3, 4]. Drawing on the research results of Cheah and Ho [5], relationship dynamics can be positive or negative. Compared with a selfish competition-oriented relationship, a positive dynamic relationship is more inclined to enhance the survival and progress of the ecosystem with an attitude of cooperation. The ecosystem becomes an open architecture that enables members to access and use resources to develop new services that can interact with and enhance existing services [6]. Openness and reciprocity can be developed to explore the functions of the entire ecosystem and each participant, which is what Pera et al. [7] describe as a cocreation service ecosystem. The cooperation of relevant participants in the process of resource integration can improve resource insufficiency and density [8, 9].

Digital media asset management refers to the use of computer technology, network technologies, database technology, mass data storage, and so forth, using scientific theories and methods through the planning, organization, storage, control, development, and utilization activities of digital media assets and the life cycle process of management and utilization activities to improve the use efficiency of assets and maximize asset value. Kurti et al. [10] applied the communities of practice approach to establish a knowledge management system and explored the methods of constructing, sharing, and using tacit and explicit knowledge in the community of practice. Lee et al. [11] proposed a cultural creativity driving industry collaborative innovation and coevolution framework, discussed how the business ecosystem is based on collaborative innovation through cooperation to achieve cooperative coevolution of different structures and directions to build the generalized innovation process at the ecosystem level, analyzed the process of cooperation in the system, and carried out exploratory research on the OTT platform. There is evidence that social media changed the dynamic interaction between organizations and consumers through the establishment of online relationships, and these dynamic channels are challenging the traditional belief of the effectiveness of one-way marketing. Exploring the diffusion of social media content within the ecological framework can improve the understanding of the existing social network service dimensions [12].

From the platform perspective, the platform ecosystem is a complex system composed of many subsystems interacting dynamically. The value of the platform ecosystem is created by all participants [13]. To a certain extent, value cocreation theory highlights the complexity of the interacting subject in the context of platform ecosystems [14]. Marketing scholars have not yet reached a consensus on the definition of platform ecosystems. Some scholars regard the platform as a component of the service ecosystem, a physical or virtual contact point that provides structural support for resource integration among participants in the service ecosystem [15, 16]. Some scholars also regard the platform as a complex service situation, which is a cross-interactive platform system [17] that promotes enterprises and customers to form higher-order resources [18].

Based on the statement above, research on business ecosystems is mainly carried out from the perspectives of value proposition, value network, value maintenance, value realization, and so forth. All these studies provide references for this study. Previously published studies also have shortcomings: they describe the key aspects of business model innovation from individual factors in the system; however, few studies have considered that the system is a collection of many factors. To date, China's digital media asset management and service patterns still need to be improved. The system dynamics approach is good at abstracting the relationship between various factors in the system, and its characteristics match the research problem. Therefore, this study is based on the business ecosystem of digital media asset management and the service pattern of the key influencing factors, using a system dynamics approach to construct a digital media asset management ecosystem model. More importantly, the model can further analyze the dynamic evolution process of content assets value increment in the model, having theoretical significance and having more important practical application value. This plays an important role in accelerating the integration of media content resources, improving management concepts, innovating service models, and expanding larger market space.

The remaining part of the paper proceeds as follows.  Section 2 combines business ecosystem thinking and intelligent digital media asset management and discusses the positioning of digital media asset management and service patterns. A system dynamics approach to construct a system dynamics model is provided in Section 3. In Section 4, the main results of the study are given. The conclusions and future research directions are outlined in Section 5.

## 2. The Positioning of Intelligent Digital Media Asset Management and Service Patterns Based on Business Ecosystem

Based on business ecosystem thinking, the digital media asset management ecosystem brings about a series of changes in digital media assets from content management and the business model to the industrial chain layout. Suppose that media organizations such as radio and television decide to promote media convergence and realize the operation of digital media asset management platforms. In that case, they need to start from the top-level design, establish a platform-based intelligent digital media asset management ecosystem, and efficiently connect the upstream, midstream, and downstream of the digital content industry chain. The value of digital media assets is maximized by connecting content resources, content production, content service, and product development.

### 2.1. Establish a Platform-Based Intelligent Digital Media Asset Management and Content Service Patterns

#### 2.1.1. Unified Digital Media Asset Management Platform

Content and platforms are the two pillars for the survival and development of the modern media industry. This makes it necessary for media organizations to establish a media assets management platform that can collect, manage, and reuse various digital contents such as broadcast and video content at the public level. It should also support the unified management of various types of digital content in content integration, content management, content sharing, content product development, and other links. Then, they enhance the ability of media organizations in content operations, vertical development of content, and diversified services. The unified management platform for digital media assets established through integration comprises media asset management centers of TV stations, radio stations, and other broadcasting and television institutions at all levels. The interaction between content providers and users is taken into account.

Today's world is a network-based, interconnected, and interdependent world. In this context, this study believes that the development of media organizations should be built based on a value network, taking new business models as benchmarks, cooperation, specialization, and provision of a multiwin content service platform as the key to success. The establishment of platform-based digital media asset management and content service patterns requires a detailed investigation and analysis of the market environment and focuses on four positioning directions: the integration and aggregation of digital media content resources in multiple directions to meet large-scale requirements; meeting the needs of the neglected part of the market and improving the value creation ability of niche markets; innovating and developing new content products and services and bringing them to the market; innovating business models, changing the competition pattern of the existing market, and creating new products and services to improve the operating efficiency of the entire market.

#### 2.1.2. Effective Intelligent Digital Media Asset Management Mode

With the digital transformation of media organizations, the value chain of the media content industry has changed, and media organizations represented by radio and television are facing challenges in management mode, copyright management, content product value evaluation, operation mode, and many other aspects. In terms of management mode, media organizations need to form an effective management mode and development methods to fully tap the existing large number of programs and materials; otherwise, the quality and quantity of the rapid creation of new programs will be restricted, thus limiting the play of competitive advantages. In terms of copyright protection, the copyright management and protection efforts of media content assets need to be further strengthened to effectively solve the copyright disputes and copyright payment problems of digital assets. In terms of the pricing of media content products, there is no industry-recognized standard for evaluating and pricing media content assets, which also restricts the large-scale marketing of programs, materials, and content products of secondary creation. Therefore, the formulation of industry evaluation standards needs to be accelerated. In terms of operation mode, with the increase in people's demand for media content, traditional media need to effectively expand the business operation mode of content products under the new media convergence competition environment, and its innovation ability needs to be improved.

Building a platform-based intelligent digital media asset management ecosystem solves the above problems with a better business model, supports the main business processes and workflows in radio and television media, and flexibly adapts to new workflows to achieve higher productivity, faster efficiency, better service, lower costs, and increased agility and adaptability of the whole system. To improve effectiveness and efficiency, ecosystems can be connected with other applications and systems, such as databases and information systems, production systems, news studio systems, automation systems, record and display systems, media resource planning systems, and copyright management systems. In addition, ecosystems should open up data to relevant members of the ecosystem through real-time visibility and information sharing. Therefore, ecosystems must provide interfaces to these systems that allow cross-platform retrieval, collection, and delivery, including the exchange of metadata and materials. Based on the digital media asset management platform, the digital media asset management ecosystem can reduce the problem of information duplication in the business, break the information silos, and promote the integration and sharing of information and content to better manage digital assets. Thus, only through an integrated solution can a harmonious and consistent digital media asset management ecosystem be achieved.

Information duplication is the first major problem, and a content management system (CMS) can be used to store all media resource information in a single repository and reduce the risk of information duplication across business units, which is an effective way to reduce maintenance costs and error rates. Completing a workflow often requires multiple attempts. When multiple systems are used to manage content information, managing content information may span different systems. If the workflow is fragmented, the system treats each iteration as a new piece of content, resulting in content data duplication. Therefore, it is important to examine the process for potential defects. This study suggests that an effective intelligent digital media asset management mode should achieve overall expansion in an evolving media environment to better pursue efficiency and value. A digital media asset management platform should establish digital governance alliances to centralize data in a managed environment, making it easily accessible to those who can determine the value of the data. Working together to address workflow duplication, data accuracy, and data consistency, actively cooperate with the statistical work of relevant content resources and reduce the duplication of information and content to better respond to the evolving digital asset management ecosystem. Information silos are the second major problem. When there is an information silo in a media organization, version selection errors tend to occur during distribution because there may be multiple versions of the same content. Using a unified digital media asset management platform for management can prevent this from happening.

Therefore, it is of great significance to perfect digital media asset management platform construction, continue to promote content asset sharing and digital governance, establish a system encouragement mechanism to solve the problem of information duplication and information silos, promote the value creation of content, lower program production costs, and improve the quality of shared data in the content database.

### 2.2. Industrial Value Chain Extension of the Digital Media Asset Management Ecosystem

#### 2.2.1. Industry Value Chain of Digital Media Asset Management Ecosystem

The value chain of the digital media content industry based on the business ecosystem emphasizes strengthening the diversity and connection among various entities, thereby enhancing the industry's competitiveness. The digital content industry is highly integrated with high-tech and cultural content elements. It refers to products or services that integrate images, text, video, voice, and other contents by means of digital high-tech. With the rapid innovation and application of digital technologies such as cloud computing, mobile Internet, big data, and artificial intelligence, the development of the content industry is more inseparable from digital content. To understand the ecological environment of digital media asset management, there is a new way of thinking about applying the theory of information ecology to the management, development, and utilization of content resources in the media content industry chain. Therefore, the industry value chain of digital media content is the primary issue that needs to be considered when studying platform-based digital media asset management ecosystems.

Because of the continuous development of media convergence in media organizations such as radio and television, the media industry within different types of value creation activity forms changed dramatically, from once upon a time an enterprise or organization, gradually dispersed to multiple enterprises or organizations to participate in activities to jointly create value in this way. The value chain of the digital media content industry consists of multiple links and multilateral groups, and there are different subjects participating in each link. These links can be divided into three parts: upstream, midstream, and downstream. The core of the upstream part is content production, involving content creators, content producers, and so forth. The midstream part is mainly content processing, distribution, and communication activities, involving traditional retail publishers, service operators, and other sales channels and communication media. The end of the downstream part is mainly the content consumers of institutional users and individual consumers. From the perspective of ecosystems, further attention should be given to the integrated development of related industries, to expand the business model to more relevant groups and lay a broader foundation for the expansion of market and profit space.

In the process of promoting digital media asset management ecosystem construction, it is necessary to use modern communication technologies and operational concepts to break through the limitations of traditional radio and television media in platforms, channels, and mobile terminals. While broadening the scope of cooperation with network operators, live video sites, software development, and other unit cooperation, they optimize the allocation structure of resources and get through all links of the industrial chain.

#### 2.2.2. Intelligent Digital Media Asset Management and Development Application Cases

By establishing a platform-based digital media asset management ecosystem, Chinese media organizations can respond to emerging broadcast and sales channels through new business models and make strategic plans. They can provide audio/video-on-demand, broadband access, short video, mobile streaming media, and copyright sales to meet the needs of new and old users. At the same time, a diversified industrial chain has been formed, including the production of multiple types of film and television content authorization products, the linkage of games, the landing of theme parks, the promotion of cultural and creative products, and the construction of parks. Content is the core competitiveness of the media industry. Media organizations represented by radio and television produce a large number of programs every day and gradually accumulate large digital media assets. Given this, most of China's provincial and municipal television stations and radio stations have established media asset systems. Taking China Central Television as an example, its media content assets have more than one million hours. In addition, the European and Latin American Language Program Center of China Media Group has established a platform-based digital media asset management ecosystem to meet international communication needs. It also built a media business integration platform to better service the Beijing headquarters of the Euler Center and their localized communication agencies distribution in Europe and Latin America. It also built a business communication chain for business interconnection and cooperation and program exchange between Euler Center headquarters and localized communication agencies, which can realize public opinion aggregation, information collection, media content production, multichannel matrix release, distributed storage, global management, and comprehensive communication data feedback services.

In recent years, television broadcasters have begun to value public access to the contents of their archives and have gradually made their archives available to researchers and the public. To explore the value and potential of its archives, the BBC has developed the BBC Programme Explorer. By using this tool, more than 200,000 programs can be retrieved more conveniently and quickly, improving the program production efficiency of the BBC staff, saving costs, and recycling media resources. The National Audiovisual Institute (INA) is a national audiovisual data agency for users worldwide which aims to collect, protect, digitize, store, and promote audiovisual data for French television and radio. INA actively explores the provision of online TV content services for the public, allowing users to pay to watch video and audio materials and access the content catalog reviewed and selected by INA and obtain program content by downloading through its own portal. Some archives actively expand the market, seeking professionals who need to reuse resources and explore new partnerships. Some archives believe that there is great potential for their capabilities and resources in the education market and choose to partner with educational publishers and platforms for massive open online courses (MOOCs), leveraging these existing channels to maximize their impact. Given the demand for online services from performing arts venues, some archives have worked with music, theatre, and opera companies to create a richer viewing experience by adding recordings of relevant content to online performing arts catalogs.

## 3. System Dynamics Model Construction of Intelligent Digital Media Asset Management

### 3.1. Analysis Framework of the Digital Media Asset Management Ecosystem

#### 3.1.1. Characteristics of Digital Media Asset Ecosystem

The main direction of digital media asset management platform value is to be supported by information technology and focused on content innovation, building media ecology through high-quality media content. Specifically, a good digital media asset management ecosystem includes not only structural design and information technology but also content strategy, political factors, behavioral factors, partnerships, market positioning, support staff, business processes, and profit models. There is much room for improvement in traditional media asset management systems. On the one hand, traditional media asset management is usually a closed system that not only lacks linkage with external resources and capabilities but also lacks an effective response to the rapid production mode of program content in the new media era. On the other hand, traditional radio and television media asset system management often ignores the importance of operation management, has insufficient understanding of the value of digital media assets, and is not strong in pioneering and innovative consciousness.

The characteristics of the digital media asset management ecosystem lie in emphasizing the integration of various types of information and content resources, emphasizing the development and evolution of the content asset management system ecological environment, and emphasizing the role and interest balance of all parties involved. If media organizations want to gain competitive advantages in the three-dimensional market competition environment, they must find their own unique value network by connecting and cooperating with ecological partners in the digital ecological community.

The core of digital media asset management is asset value management, which is reflected in the value-added management processes of asset value recognition, protection, development, and pricing. In the digital media assets of media organizations represented by radio and television, not only do video and audio have value, but also the information value contained in these media contents has a great potential for mining. In the digital media asset management ecosystem, value creation is accomplished based on the digital media asset management platform, which is composed of media asset management centers of TV stations, radio stations, and other broadcasting and television institutions at all levels, and related subjects.

In the value creation process of digital media asset management ecosystem, it is necessary not only to participate in multiple subjects but also to solve the problems of effective management and redesign and realize the value integration of digital media content in different media organizations. This can play a large role in content integration, content innovation, content flow, and content utilization. In the convergence media environment, some media organizations have established digital content asset databases to meet the growing user demands. The advantage is that, in addition to continuously promoting the content data sharing and establishing a system encouragement mechanism, it can also reduce the cost of program content business production and improve the quality of shared data in the content databases to create content value. On this basis, the digital media asset management ecosystem can be better integrated into market analysis, advertising, copyright management, creative services, production, sales, and distribution. To broaden revenue channels, expand markets, and enhance user stickiness, media organizations actively explore the transformation of media platforms and try to speed up the effective flow of content on different media platforms through new technologies and marketing strategies. An effective flow is not simply uploading and distributing the content, especially the programs on the big screen, to various platforms and channels. Instead, the content needs to be adjusted according to the characteristics of different platforms and channels.

#### 3.1.2. Structure Analysis of Digital Media Asset Management Ecosystem

According to the characteristics of the digital media asset management ecosystem, this study further analyzes its structural levels and proposes a platform-based digital media asset management ecosystem, as shown in Figure 1. Within a specific time and space, a complete ecosystem is formed by stakeholders, such as digital media content assets, content providers, consumers, and content asset value realization environments, which jointly affect the realization effect of digital media asset value. Specifically, this system is a digital media asset management ecosystem consisting of digital media asset management subjects, the digital media asset management platform, digital media asset management environments, and digital media asset management technologies. There is a competitive and cooperative relationship between relevant industrial subjects involved in digital media content management. Digital media asset management subjects, the digital media asset management platform, and digital media asset management environments continue to exchange and feedback of content and information. With the help of information flow, capital flow, workflow, and other functions, they form an open and dynamic system.

The digital media asset management platform is a unified management platform formed by integrating media asset management centers of radio, film, and television institutions, which provides the content resources, media asset management system, and service mode of media asset management. The platform mainly includes digital media content resources, content integration, innovation activities, content flow, content utilization, and cooperation performance distribution factors [19]. The digital media asset management environment mainly includes the policy environment, legal environment, market environment, convergence industry, economic environment, and other external environments, as well as the content operation internal environment of the digital media asset management platform. Digital media asset management technologies mainly include platform construction, technical support, and other influencing factors. The digital media asset management ecosystem brings new market opportunities and business models for the content industry. In the future business ecology of digital media assets, the platform-based digital media asset management ecosystem can be developed by deepening strategies related to vertical growth within the same industry on the one hand. On the other hand, it can also be developed by connecting different industries with expansion strategies related to horizontal growth [11].

### 3.2. Establishment of a System Dynamics Model

#### 3.2.1. Model Suitability Analysis

Business models of digital media asset management are dynamic [20]. Therefore, the digital innovation of business models becomes imperative for survival in the ever-changing ecosystem. Digital media asset management ecosystem value creation is a dynamic and complex process in which multiple subjects develop and utilize the digital content of the assets of media organizations and apply the value to specific problems. The development of the digital media asset management ecosystem is influenced by internal and external factors, forming an interactive information flow that is a nonlinear system. At the heart of the digital media asset management ecosystem is the constant flow of content assets between media organizations, which can be accumulated, reused, and restructured to create new content to better tap its potential value. In addition, the inventory and value of digital media content continue to grow, and there are multiple feedbacks, which are in line with the basic research conditions of system dynamics.

In view of this, this study adopts a system dynamics approach to construct a system dynamics model of the digital media asset management ecosystem. Based on the simulation analysis of digital media asset management and service innovation behavior, it discusses how digital media asset management can promote the value-added of content assets. Therefore, the logical relationship between the internal elements of the system and its running rules will be more intuitively and clearly identified to better promote the content flow and value creation of the digital media asset management ecosystem and innovate digital media asset management and service modes [21].

System dynamics (SD), proposed by Jay W. Forrestrer in 1956 and published in 1958, is an effective tool for studying complex information feedback systems through differential equation analysis and further analyzing social science problems. Scholars increasingly use SD as a research method [22]. SD modeling is suitable for simulating and examining complex and dynamic systems and supporting long-term, strategic decision-making [23]. For example, some scholars use the system dynamics method to study the influence of different Internet application environments on knowledge transfer between enterprises from the perspectives of Internet tools, Internet platforms, and Internet resources [24]. Some scholars use system dynamics and agent-based modeling to represent intangible process asset characterization [25]. In the digital media asset management ecosystem, under the background of a convergence media environment, the impact of digital media content between different media organizations to effectively manage, and the values of many factors, the relationship between these factors is more complex. Thus, the system dynamics method can be used to parallelize the influencing factors and abstract the relationship between influencing factors.

An ecosystem composed of digital media asset management subjects and digital media asset management environments has a relatively clear system boundary. The flow of digital media content assets within the system has a certain predictability and regularity, rather than being random and unstable. Therefore, this study comprehensively constructs a system dynamics model and analyzes the dynamic evolution process of content assets value increment in the digital media asset management ecosystem by using causal charts and flow charts for simulation analysis.

#### 3.2.2. The Causal Model and Main Feedback Loops

This study constructs a causal model of value creation in the digital media asset management ecosystem, as shown in Figure 2. According to the system feedback represented by the loops in the causal model in Figure 2, we can find the main feedback loops that reflect the core elements of digital content asset value realization, such as technical input, platform operation input, and content asset integration and utilization.

#### 3.2.3. Model Assumptions and System Dynamics Flow Chart

To standardize the issues raised in this study and clarify the premises and conditions for the operation of the digital media asset management ecosystem, the following basic assumptions are proposed based on the analysis of the value chain of the content industry and the basic framework of the digital media asset management ecosystem constructed in Section 3.1.

1. Content asset management conducted by media organizations based on the digital media asset management platform is a continuous and gradual value creation process consisting of key activities such as content asset acquisition, integration, innovation, flow, utilization, and value realization.
2. The input end of the system refers to the programs, materials, and other media content resources provided by content providers for media organizations. In contrast, the output end of the system refers to the competitive advantages obtained by media organizations based on digital media content asset management, which is mainly measured by the income of platform participants.
3. This model does not consider the system behavior changes caused by unpredictable emergencies or accidental factors such as major policy changes and natural disasters.

Based on the model's assumptions and the causal model in Figure 2, the corresponding system flow chart is constructed in this study, as shown in Figure 3. The model contains 4 state variables, 5 rate variables, 30 auxiliary variables, and 3 constants, as shown in Table 1. The system flow chart reflects the interactive relationship, system structure, and dynamic characteristics of various factors in the process of value realization of the digital media asset management ecosystem, which has positive significance for media organizations to carry out innovative activities in digital media asset management.

#### 3.2.4. Model Equation Design and Parameter Explanation

In the process of building the system dynamics model, attention should be given to the causal relationship of the model to reflect the real dynamic behaviors of the system and avoid the one-sided pursuit of unnecessary complex models [26]. The establishment of system dynamics equations is an essential step in the modeling process. The equations can quantitatively process the variables in the system and quantitatively analyze the operation mode of the digital media asset management ecosystem.

To simplify the study, the equations are designed and explained based on the existing research and causal analysis and combined with the actual situation of digital media asset management. The main system dynamics equations and parameters were determined as follows:

1. The stock of content assets on the platform = INTEG (the increase of the number of content assets, 1000);
2. Digital content assets value increment = the number of content assets utilized *∗* average content asset price;
3. Profitability of platform participants = INTEG (platform participants' income - platform participants' input, 1000);
4. The number of content assets utilized = INTEG (content assets utilization increment, 1);
5. Content assets utilization increment = the amount of content asset flow *∗* content asset utilization rate;
6. The amount of content asset flow = the amount of content asset innovation *∗* content asset flow rate;
7. The amount of content asset innovation = content asset innovation rate *∗* the amount of content asset integration;
8. The amount of content asset integration = (content asset integration capability + degree of sharing of content asset) *∗* the stock of content assets on the platform *∗* 0.1;
9. The amount of content assets increase = the stock of content assets on the platform *∗* content assets acquisition rate + the amount of content asset innovation;
10. Digital media asset management investment = platform participants' income *∗* digital media asset management investment rate;
11. Digital media asset management investment rate = WITH LOOKUP (time, ([(0, 0) (24, 10)], (0, 0.2), (24, 0.25)));
12. The intensity of the platform operation input = LN (profitability of platform participants) *∗* 0.2;
13. The intensity of digital media asset management technology input = LN (profitability of platform participants) *∗* 0.15;
14. The value positioning ability of platform participants = INTEG (the cognition degree of platform participants to user requirements, 500);
15. Digital media asset management capability = the intensity of manpower input *∗* 0.3 + the intensity of the platform operation input *∗* 0.4 + the intensity of digital media asset management technology input *∗* 0.3;
16. Stakeholders' willingness to collaborate = RANDOM UNIFORM (0.1, 1, 24) *∗* the rationality of cooperation performance distribution *∗* value realization environment *∗* 0.1;
17. Relevant industry support = WITH LOOKUP (time, ([(0, 0) (24, 1)], (0, 0.1), (24, 0.6))).

## 4. Simulation Results

### 4.1. System Boundary

This paper aims at the digital media asset management ecosystem based on the business ecosystem. On this basis, it analyzes the changing characteristics of digital media asset management to realize the value increment of content assets. In determining causality and the construction of the model, the time problem and the important variables closely related to the research topic are considered. The less important endogenous variables and exogenous variables with less influence are considered to clarify the research question.

### 4.2. Simulation Analyses

In this study, Vensim PLE software is used for simulation analysis. Assuming that the initial value of the content asset stock is 1000, the simulation duration is set to 24 months. The content asset integration capability, the number of content assets utilized, the stock of content assets on the platform, the quality of content products and services, and the digital content assets value increment are selected as test objects. The simulation results of the dynamic evolution process of the digital media asset management ecosystem are shown in Figure 4.

As seen from the simulation results, the content asset integration capability, the number of content assets utilized, the stock of content assets on the platform, the quality of content products and services, and the digital content assets value increment tend to increase gradually with time.

The content asset integration capability is the key control point of the digital media asset management platform. Media organizations and value nodes integrate and develop resources through the platform to support the system's efficient operation. In the digital media asset management ecosystem, business process management capabilities, the degree of standardization of content assets, stakeholders' willingness to collaborate, and the rationality of cooperation performance distribution all affect the content asset integration capability, which leads to changes in the amount of content asset innovation and ultimately affects the digital content assets value increment.

In addition, the improvement of the content asset integration capability has a positive impact on the number of content assets utilized. On the one hand, with the gradual maturity of the market, content asset innovation rate, content asset flow rate, content asset utilization capability, and relevant industry support are constantly improving, resulting in an increase in the amount of content asset innovation, which increases the amount of content asset flow. On the other hand, the value realization environment, content asset utilization capability, and other factors affect the utilization rate of content asset and the number of content assets utilized.

Content assets are the resource base of value creation activities of broadcasting and television media, and the stock and quality of content assets are the keys to determining the behavior of the entire digital media asset management ecosystem. With the development of increasingly innovative program content, the amount of content asset innovation continues to increase. Then the stock of content assets on the platform increases, making the number of content assets utilized and value increment present an increasing trend.

The quality of content products and services is a key factor affecting user satisfaction, as well as a comprehensive reflection of the intensity of the platform operation input, the intensity of manpower input, the value positioning ability of platform participants, and the intensity of digital media asset management technology input.

The digital media assets value increment is a measure of the efficiency of the whole digital media asset management ecosystem and the level of content product and service. At the beginning of system operation, the digital content asset value increment is at a low level due to the low content asset utilization rate and digital media asset management capability. In the process of system value creation, the amount of content asset flow and content asset utilization rate are constantly improved so that there are more available content assets in the system, thus providing users with richer content products and services, promoting the quality of content products and services, and further increasing the value of content assets.

According to the analysis above, the system dynamics model of the platform-based digital media asset management ecosystem model constructed in this study can reflect the trend of the dynamic change process of digital media assets value increment, indicating that the model is reasonable and effective.

### 4.3. Sensitivity Analysis

Sensitivity analysis is used to analyze the sensitivity of the system to numerical adjustment by observing the degree of curve change to change the parameters in the model. In this study, the sensitivity of the model is analyzed by gradually changing the values of the intensity of digital media asset management technology input and the intensity of the platform operation input in the model.

The corresponding curve of the original plan is noted as current1. Based on the original plan to improve the technology input rate of the management platform and increase the value of the parameter, the intensity of digital media asset management technology input was increased by 10%, 20%, 30%, 40%, and 50%, respectively, with each new curve noted as current2, current3, current4, current5, and current6. The digital content assets value increment is shown in Figure 5. Figure 5 shows that the intensity of digital media asset management technology input significantly impacts the digital content assets value increment, and the two are positively correlated. With the rapid development of information technology in the external environment, media organizations should strengthen the introduction of digital media asset management technologies and provide the necessary technical support for the normal operation of the digital media asset management platform. TV stations, radio stations, film and television companies, and other broadcasting and television institutions often have their own digital content assets database. Increasing the intensity of digital media asset management technology input can promote the degree of sharing of content assets between radio, film, and television institutions, thereby improving the degree of standardization of content assets and the rationality of cooperation performance distribution and further enhancing the ability of content asset resource integration. With the help of an effective intelligent digital media asset management mode, the effectiveness of digital media management can be enhanced through consolidation, integration, and adoption of new IT equipment and business processes so that the IT equipment and business process of the next level department of media organization can be quickly integrated into the mainstream system of the next level. Content asset integration and business process reengineering can expand the scope of information and content sharing by constructing the cloud service platform of the broadcasting and television content industry and have a positive impact on the degree of digital media asset integration. In addition, the standardization of media content assets needs to fully consider data structure, data interface, data storage, data distribution, production processes, and so forth. The deeper the degree of standardization of content assets is and the more standardized the format is, the easier the data transformation between various systems will be. It will promote the integration of digital content resources in the digital media asset management platform.

In the digital media asset management ecosystem, the intensity of the platform operation input is the key to digital media asset management. The corresponding curve of the original plan is noted as current1. Based on the original plan and increasing the value of the parameter, the intensity of operation input was increased by 10%, 20%, 30%, 40%, and 50%, respectively, with each new curve noted as current1, current2, current3, current4, current5, and current6. The digital content assets value increment is shown in Figure 6. Figure 6 shows that increasing the intensity of platform operation input positively impacts the digital content assets value increment. On the one hand, radio and television media should strengthen the operational input of the digital media asset management platform to promote content asset integration and development capability and form effective business processes and development methods to fully tap the existing large number of programs and materials. This will improve the quality and quantity of new programs created quickly and give full play to their competitive advantages. Ultimately, this will increase the value creation level in the digital media asset management ecosystem. Using an effective intelligent digital media assets management mode carries on the effective management between radio and television media to design and realize the value of integration. For example, in the market analysis, advertising, rights management, innovative services, production, sales, and distribution are aspects of better integration, thus reducing the pressure of the radio and television media from competition, innovation, and cost reduction. On the other hand, the construction of a digital media asset management platform should be strengthened. Text, pictures, audio, and video resources are collected with the help of intelligent technologies to achieve audio and video resources in the whole management process while supporting a variety of efficient retrievals. In addition, according to the characteristics of business and user groups, personalized services are provided to meet the business needs of distribution and invocation on multiple channels and to provide digital and standardized processing services. Based on the intelligent digital media assets management mode, it can solve the problems of the content and technology of digital assets in media organizations and workflow discontinuity to improve the operational efficiency of media and reduce costs. In addition, establishing the copyright management system of digital assets based on the platform can make copyright management play a role more quickly and effectively by adopting new technologies and methods.

## 5. Conclusions

Based on the business ecosystem, this study takes China's broadcasting and television media organizations as the research object, deeply exploring the value creation process accomplished based on the digital media asset management platform through theoretical analysis methods and simulation analysis. First, the positioning of intelligent digital media asset management and service patterns is comprehensively and systematically analyzed. Then, the key influencing factors of intelligent digital media asset management and service patterns based on the business ecosystem are explored. The focus is on establishing a platform-based digital media asset management ecosystem, which is continuously deepened in terms of the value chain. Second, the paper discusses the characteristics and structure of the digital media asset ecosystem and puts forward the basic framework of intelligent digital media asset management from the perspective of content asset value management elements. Finally, the system dynamics model of intelligent digital media asset management is constructed using the system dynamics simulation method, which can better demonstrate the value creation factors of the digital media asset management ecosystem and the system operation rule. This study offers important insights for media organizations to manage digital media assets effectively and achieve a greater value of the content assets.

The simulation results show that the content asset integration, content asset innovation, content asset flow, content asset utilization, digital media asset management technology input, platform operation input, and value realization environment all act on the value creation of digital media content assets. The content asset integration capability, the number of content assets utilized, the stock of content assets on the platform, the quality of content products and services, and the digital media assets value increment will continue to grow with the system's operation. To fully realize the value of digital media content assets, media organizations should attach great importance to the value management of content assets and strengthen digital media asset management technology innovation, platform operation, and process management to improve the utilization of content asset and the quality of content products and services. Strengthen the division of labor and collaboration among multiple subjects and encourage relevant industry groups to participate in content cooperation to increase content asset utilization capability.

At present, there are few studies using system dynamics to analyze digital media asset management. This paper presents an unprecedented approach based on system dynamics simulation that provides effective strategic decisions for media organization decision-makers. Stakeholders will be able to use a simulation tool to understand the elements of the digital media asset management ecosystem's influence on content assets value increments, emphasizing the importance of effective digital media asset management. However, due to the complexity of the value realization of digital media asset management and the particularity of media content products, some indicators are difficult to quantify. The value realization of the digital media asset management ecosystem is only an abstract process. Therefore, the empirical analysis of the model based on real data is not carried out in this study, only considering the key factors and simplifying some variables of content assets management. Future studies need to further study the complex model containing more comprehensive influencing factors, verification of the research model, and the conclusions of this paper.

## Figures and Tables

**Figure 1:** Basic framework of the digital media asset management ecosystem.

**Figure 2:** Causal chart of value creation in the digital media asset management ecosystem.

**Figure 3:** Value creation flow chart of the digital media asset management ecosystem.

**Figure 4:** Simulation results.

**Figure 5:** Adjusting the results of the sensitivity analysis of the intensity of technology input.

**Figure 6:** Adjusting the results of the sensitivity analysis of the intensity of the platform operation input.

**Table 1:** Variables in the system flow chart.

Variable type	The number of variables	Variable names
State variable	4	The stock of content assets on the platform, the number of content assets utilized, profitability of platform participants, the value positioning ability of platform participants
Rate variable	5	The increase of the number of content assets, content assets utilization increment, platform participants' income, platform participants' input, the cognition degree of platform participants to user requirements
Auxiliary variable	30	Degree of sharing of content asset, the amount of content asset integration, the amount of content asset innovation, content asset innovation rate, the amount of content asset flow, content assets acquisition rate, content asset flow rate, content asset utilization rate, content asset utilization capability, relevant industry support, digital content assets value increment, content asset integration capability, degree of standardization of content assets, business process management capabilities, digital media asset management capability, the rationality of cooperation performance distribution, digital media asset management investment, digital media asset management investment rate, stakeholders' willingness to collaborate, the intensity of the platform operation input, the intensity of digital media asset management technology input, the quality of content products and services, user satisfaction, user requirements, value realization environment, technology environment, policy environment, social environment, media organization environment, average content asset price
Constants	3	Platform participants' other incomes, platform participants' other inputs, the intensity of manpower input

## Data Availability

The data used to support the findings of this study are included within the article.
